# Anti-Inflammatory Effects of the Chinese Herbal Formula Sini Tang in Myocardial Infarction Rats

**DOI:** 10.1155/2014/309378

**Published:** 2014-03-03

**Authors:** Jiangang Liu, Karoline Peter, Dazhuo Shi, Lei Zhang, Guoju Dong, Dawu Zhang, Heimo Breiteneder, Rudolf Bauer, Johannes Jakowitsch, Yan Ma

**Affiliations:** ^1^Center of Cardiology, Xiyuan Hospital, China Academy of Chinese Medical Sciences, No. 1 Xiyuan Caochang, Haidian District, Beijing 100091, China; ^2^Molecular Research in Traditional Chinese Medicine Group, Department of Pathophysiology and Allergy Research, Vienna General Hospital, Medical University of Vienna, Waehringer Guertel 18-20, 1090 Vienna, Austria; ^3^Department of Pharmacognosy, Institute of Pharmaceutical Sciences, University of Graz, Universitaetsplatz 4/I, 8010 Graz, Austria; ^4^Clinical Division of Cardiology, Department of Internal Medicine II, Vienna General Hospital, Medical University of Vienna, Waehringer Guertel 18-20, 1090 Vienna, Austria

## Abstract

The aim of this study was to evaluate the anti-inflammatory profiling of the Chinese herbal formula Sini Tang (SNT) in myocardial infarction (MI) rats. SNT, a decoction consisting of four herbs: *Aconitum carmichaelii*, *Cinnamomum cassia*, *Zingiber officinale*, and *Glycyrrhiza uralensis*, was characterized as a remedy to treat syndromes corresponding to heart failure and MI in China. Potential biomarkers, which reflect the extent of myocardial necrosis and correlate with cardiac outcomes following MI, such as atrial natriuretic peptide (ANP), high sensitivity C-reactive protein (hs-CRP), and proinflammatory cytokines such as tumor necrosis factor-**α**, interleukin-6, and interleukin-1**β** (TNF-**α**, IL-6, and IL-1**β**) were determined in plasma, serum, and in myocardial tissue of MI rats after treatment with SNT. Our data indicate that SNT decreased significantly the levels of hs-CRP, TNF-**α**, IL-6, and IL-1**β** in MI rats. SNT decreased the expression of ANP levels in plasma and increased the vascular active marker nitric oxide, which limits vascular inflammation. In addition, SNT could decrease the expression of endothelin-1 levels in rat plasma post-MI. Our data suggest that the Chinese herbal formula SNT has the potential to improve cardiac function after MI. SNT may be a candidate for treating MI and its associated inflammatory responses.

## 1. Introduction

Heart failure (HF) is a critical disease. Currently 26 million people are suffering from HF worldwide, one quarter of them in Europe [1]. One of the major causes of HF is myocardial infarction (MI). Every sixth man and every seventh woman in Europe died from MI [2]. MI is associated with an inflammatory reaction, which is a prerequisite for healing and scar formation [3, 4]. Inflammatory markers such as interleukin-6 (IL-6), interleukin-1*β* (IL-1*β*), high sensitivity C-reactive protein (hs-CRP), and tumor necrosis factor-*α* (TNF-*α*) reflect the extent of myocardial necrosis and correlate with cardiac outcomes following MI [5–7].

Traditional Chinese medicine (TCM) has been used in China for centuries for treatment of cardiac disease and is now attracting interest in Western countries as a source of alternative or complementary therapies due to its reputed effectiveness, low cost, and relative absence of side effects. Previous studies provided scientific evidence to support the use of Chinese herbal medicine for treating MI and HF [8–13]. A TCM Sini Tang decoction (SNT), which consists of four Chinese medical herbs, the root of Sichuan aconite (*Aconitum carmichaelii* Debeaux, Ranunculaceae), the bark of Chinese cinnamon (*Cinnamomum cassia* J. Presl., Lauraceae), the rhizome of ginger (*Zingiber officinale* Roscoe, Zingiberaceae), and the root of Chinese licorice (*Glycyrrhiza uralensis* Fisch. ex DC. Fabaceae) [14], was used in preliminary and previous studies in a MI rat model [15, 16] (Table 1).

The crude aconite contains the highly toxic diester-diterpenoid alkaloids aconitine, hypaconitine, and mesaconitine. Our previous results indicated that SNT is suitable and safe for the rat model and has the potential to improve early ventricular remodeling and cardiac function after MI. SNT reduced collagen matrix accumulation in the serum and in the myocardial tissue, which is associated with a significant improvement in systolic function. Furthermore, SNT decreased the expression of Toll-like receptors (TLRs) levels in the myocardial tissue. TLRs belong to a group of type I transmembrane receptors with endogenous and exogenous ligand binding ability to stimulate innate and adaptive immune responses and induce immune and inflammatory cytokines IL-6, TNF-alpha, and other gene transcriptions and protein expressions [17–20].

In this study we aimed to confirm these preliminary observations by evaluating a number of potential biomarkers and proinflammatory cytokines as well as atrial natriuretic peptide (ANP), the potent vasoconstrictor endothelin-1 (ET-1), and the vascular active marker nitric oxide (NO), which limits vascular inflammation and plays an important role in cardiac remodeling and wound repair after MI [21–24]. ANP conveys the cardiac protective properties of vasodilation, inhibition of cardiomyocyte hypertrophy, cardiac fibroblast proliferation, collagen synthesis, and enhanced lipolysis [25]. ANP and other natriuretic peptides are the gold standard biomarkers in determining the diagnosis and prognosis of HF following MI [26]. During acute myocardial infarction, ET-1 enhances myocardial necrosis and arrhythmogenesis but seems to exert a favorable effect on subsequent infarct healing and early ventricular remodeling [27]. Thus ANP, ET-1, and NO were measured and evaluated in rat plasma and serum in this study.

Compared to our previous studies we optimized the dosage of administration by using a low as well as a high dose of SNT in this study. We also used fosinopril sodium which is indicated for the treatment of HF [28, 29] and decreases the inflammatory response after MI [30] as a positive control.

## 2. Materials and Methods

### 2.1. Animals

All animal experiments were approved by the Administrative Committee of Experimental Animal Care and Use of China Academy of Chinese Medical Sciences (CACMS, Permit number CACMS/20100322) and conformed to the National Institute of Health Guide for the Care and Use of Laboratory Animals [31].

We used 90 (50% male and 50% female) Sprague-Dawley rats (180–200 g) provided by the Vital Laboratory Animal Technology Company (Beijing, China) for this study. Rats were acclimatized with a 12/12 hours light/dark cycle at a controlled room temperature of 23–25°C and a humidity of 50–70%, and rats were allowed free access to food and water for seven days before use.

### 2.2. Drugs and Reagents Information

Chemical standards of aconitine, mesaconitine, and hypaconitine were purchased from PhytoLab GmbH, Germany. Fosinopril sodium (FS) (10 mg/tablet) was supplied by Sino-American Shanghai Squibb Pharmaceutical Co., Ltd. (China). Atrial natriuretic peptide (ANP) Kit, total nitric oxide (NO), and endothelin 1 (ET-1) were purchased from GBD Ltd., USA. Interleukin-1*β* (IL-1*β*), interleukin-6 (IL-6), high sensitivity C-reactive protein (hs-CRP), and tumor necrosis factor-*α* (TNF-*α*) Kits were provided by R&D systems (USA). Coomassie blue protein assay Kit was offered by Nanjing Science and Technology Co., Ltd. (China). The Two-step Immunohistochemical Detection Kit was produced by Zhongshan Golden Bridge Biotechnology Co., Ltd. (Beijing, China).

### 2.3. Preparation of SNT Decoction

SNT (0.5 g/g extract/crude drug) including processed* Glycyrrhiza uralensis*, processed *Aconitum carmichaelii*, *Zingiber officinale,* and *Cinnamomum cassia* was prepared at the Pharmacy Department of Xiyuan Hospital, China Academy of Traditional Chinese Medicine (Beijing, China). Aconite was cut into small pieces before use. Herbs were soaked in sterilized drinking water (500 mL) for one hour in a clay pot at room temperature and cooked to boiling. The decoction was performed twice by cooking gently for 30 min each. The two obtained decocts were combined, filtered, and stored at 4°C before administration to rats [16].

### 2.4. Quality Control of SNT by HPLC

HPLC analysis of SNT decoctions was developed during this study using an agilent 1100 series LC system equipped with a Hypersil BDS RPC-18 column (100 × 3 mm; particle size 3 mm, Agilent, Germany) as described by Peter et al. [16]. A mixed standard solution of aconitine (160 *μ*g), mesaconitine (150 *μ*g), and hypaconitine (230 *μ*g) in 1 mL acetonitrile/H_2_O (80 : 20) was prepared. The mobile phase was a mixture of buffer A (an aqueous buffer, pH3, containing 15 mM ortho-phosphoric acid and 1.5 mM tetrabutylammonium hydroxide) and buffer B (0.01% formic acid in acetonitrile). Buffer A and buffer B were used for gradient elution (5–24.4% of buffer B at 0–11 min, 24.4–26% of buffer B at 11–17 min, 26–40% of buffer B at 17-18 min, 40–100% of buffer B at 18-18.1 min, and 100% of buffer B at 18.1–23 min). The injection volume was 5 *μ*L and the flow rate was kept at 0.5 mL/min at 25°C. The detection wavelength was set at 203 nm. The content of aconitine, hypaconitine, and mesaconitine samples was calculated according to Csupor et al. [32].

### 2.5. MI Model of Rats

Acute myocardial infarction (AMI) was induced in both male and female rats by left anterior descending artery (LAD) ligation. The surgical procedures were performed using the well-established technique [33, 34]. These experiments were carried out strictly in accordance with the recommendations in the national legislation of China and performed at the Center of Animals Laboratory of the Beijing Xiyuan Hospital, China Academy of Chinese Medical Sciences. All surgeries were performed under diethyl ether anesthesia and all efforts were made to minimize suffering. Rats were anesthetized with diethyl ether and placed in a supine position on a table for the operations. The left anterior descending artery (LAD) was occluded as described by Dietl et al. [15]. To prevent infection rats were given penicillin (40.000 units) after the operation for 3 days. Sixty surviving infarct rats were randomly divided into five groups (Table 2). The oral administration of the drugs began two days after AMI-induction. SNT and FS, an angiotensin converting enzyme (ACE) inhibitor as a positive control, were diluted with distilled drinking water and administered orally in a volume of 10 mL/kg body weight once every morning for 4 weeks.

### 2.6. Echocardiography Assessment

Echocardiography was performed 30 days after surgery according to the method described by Yin et al. [35]. Ten rats from each group were anesthetized by intraperitoneal injection of ethyl carbamate (6 mL/kg). After cleaning the rat chest the cardiac short axis (papillary level), left ventricle end-diastolic dimension (LVDd), and left ventricle end-systolic dimension (LVDs) were measured using an ATL HDI-5000 Diagnostic Ultrasound System (Philips Ultrasound Inc., China). The ejection fraction (EF) was calculated from the left ventricle end-diastolic volume (LVEDV) and the left ventricle end-systolic volume (LVESV) as EF% = [(LVEDV − LVESV)/LVEDV] × 100. The data calculations were performed using a single-blind method [36, 37].

### 2.7. Measurement of Myocardial Infarct Size (IS)

The pathological slice was photographed in microdistance using a Canon IXUS 90IS digital camera. The microscopic color image processing system (DpxView Pro, Korea) was used to calculate the left ventricular IS (%, myocardial infarction area/left ventricular area × 100) by an investigator who was blinded to the identity of the pathological slice as described by Takagawa et al. [38].

### 2.8. Collection of Blood and Tissue Samples

After four weeks, the anesthetized rats were sacrificed. Blood samples were taken from the left ventricle (LV) cavity and centrifuged at 3000 rpm for 15 min. Plasma and sera were obtained and conserved at −80°C for further analysis. The heart tissue were collected, weighed, and randomly assigned. One heart of each group was stored at −80°C for ELISA.

### 2.9. ELISA Assay of Serum, Plasma and Heart Tissue

Five of the twelve frozen heart tissue samples of each group were randomly picked. The heart sections were weighed and 300 mg of each sample was cut into small pieces and 1 mL of saline solution was added. After homogenization on ice, samples were centrifuged and the supernatants were stored at −80°C for analysis. ELISA tests were performed strictly according to the instructions. The protein concentration of each tissue sample was measured with the BCA (bicinchoninic acid) Protein Assay Kit (Thermo Fisher Scientific Inc., USA).

The following biomarkers, known to be involved in the process of cardiac remodeling, were determined by ELISA [39, 40]. Functional index ANP, proinflammatory cytokines IL-6, IL-1*β*, and TNF-*α*, inflammatory biomarker hs-CRP, and vascular active markers ET-1 and NO were measured in plasma, serum, and myocardial tissue samples according to the manufacturer's instructions.

### 2.10. Statistical Analysis

Data were tabulated and presented as mean ± standard deviation, and the significance of changes was assessed with one-way repeated measures analysis of variance (ANOVA). All results were tested on normal distribution by aid of One-Sample Kolmogorov-Smirnov Test. Bonferroni's Holm test was followed for multiple comparisons. One-way ANOVA Tukey HSD test was used for pairwise multiple comparisons. A value of *P* < 0.05 was considered statistically significant. Data were analyzed using the Statistical Package for the Social Sciences (SPSS Inc., Chicago, USA).

## 3. Results

### 3.1. Quality Control of SNT by HPLC

The retention times of HPLC measurement of SNT decoction and the standards mixture of aconitine, mesaconitine, and hypaconitine were under the same chromatographic conditions (Figure 1). However, no aconitine, mesaconitine, and hypaconitine were detected in the SNT decoction. SNT is suitable and safe for the rat model used in this study.

### 3.2. Effects of SNT on Echocardiography

Four weeks after MI, ultrasound echocardiography showed a significant increase of the left ventricular dimension at end diastole (LVDd) and the left ventricular dimension at end systole (LVDs) in the model group (6.24 ± 0.72 mm versus 3.29 ± 0.81 and 6.44 ± 1.59 mm versus 0.91 ± 0.20, *P* < 0.05) compared to the sham group. The FS and SNT treatment groups exhibited significantly decreased LVDs versus the sham group (FS: 3.81 ± 1.21 mm, SNT-LD: 4.95 ± 1.95 mm and SNT-HD: 3.74 ± 1.47 mm, *P* < 0.01). The FS treatment group exhibited significantly decreased LVDd (4.45 ± 1.28 mm versus 3.29 ± 0.81 mm, *P* < 0.01). The SNT treatment groups also showed decreased LVDd versus the sham group (SNT-LD: 5.37 ± 1.78 mm and SNT-HD: 4.87 ± 1.47 mm, *P* > 0.05), but not significantly. The left ventricular ejection fraction (EF) was significantly lower in the model group compared to the sham group (55.48 ± 12.89% versus 93.32 ± 2.94%, *P* < 0.01). The FS and SNT treatment groups showed an improved left ventricular function of the EF compared to the sham (FS: 78.03 ± 10.70%, SNT-LD: 69.69 ± 13.9%, *P* < 0.05 and SNT-HD: 77.83 ± 12.32%, *P* < 0.01) and model groups (FS and SNT-HD: *P* < 0.01, SNT-LD: *P* < 0.05). SNT treatment improved the cardiac function by increasing the EF by 23.63% (difference between sham group: 93.32% and SNT-LD: 69.69%), (Table 3 and Figure 2).

### 3.3. Effects of SNT on Infarct Size

The infarct size (IS) obtained using the midline length measurement is shown in Table 3. The IS values from the FS, SNT-LD and SNT-HD groups (23.91 ± 7.99 mm^2^, *P* < 0.01, 31.25 ± 10.68 mm^2^ and 27.81 ± 10.33 mm^2^, *P* < 0.05) were significantly smaller than from the model group (38.04 ± 8.35 mm^2^).

### 3.4. Effects of SNT on ANP

In comparison with the sham group, the plasma ANP levels of rats in three treatment groups were decreased after four weeks (FS: 222.26 ± 80.25 ng/L and SNT-LD and SNT-HD: 224.82 ± 80.19 ng/L and 189.05 ± 49.96 ng/L versus the sham group: 250.00 ± 21.32 ng/L). In comparison with the model group, the SNT-HD group showed more reduction of the ANP content (SNT-HD versus model group: 367.34 ± 43.20, *P* < 0.01). The data are shown in Table 4 and Figure 3.

### 3.5. Effects of SNT on ET-1 and NO

Four weeks after ischemia the ET-1 levels of the treatment groups were decreased compared to model group (FS: 166.15 ± 9.01 ng/L, SNT-LD: 166.74 ± 7.70 ng/L, and SNT-HD: 158.49 ± 9.97 ng/L versus model group: 171.09 ± 13.17 ng/L). In comparison to the model group the NO levels of all treatment groups were increased (FS: 53.78 ± 6.24 *μ*mol/L, SNT-LD: 53.06 ± 11.54 *μ*mol/L, and SNT-HD: 64.85 ± 8.74 *μ*mol/L versus model group: 48.18 ± 10.14 *μ*mol/L). The SNT-HD group showed a significant difference (*P* < 0.05) in the NO level compared to model group. The data are shown in Table 4 and Figure 3.

### 3.6. Effects of SNT on Serum and Myocardial Tissue Levels of Inflammatory Factors

The levels of inflammatory biomarker and cytokines hs-CRP, IL-6, IL-1*β*, and TNF-*α* in rat serum and myocardial tissue were decreased in the treatment groups (Table 5 and Figure 4). The treatment groups showed a significant difference in the level of hs-CRP in comparison to the model group (FS: 5.02 ± 0.71 mg/L, SNT-LD: 3.94 ± 0.61 mg/L, and SNT-HD: 3.97 ± 0.77 mg/L versus model group: 6.71 ± 0.70 mg/L, *P* < 0.01). The treatment groups showed a decrease in the level of IL-6 compared to model group (FS: 210.60 ± 38.83 ng/L, SNT-LD: 196.81 ± 22.68 ng/L, and SNT-HD: 202.55 ± 37.37 ng/L versus model group: 240.65 ± 27.80 ng/L). The levels of TNF-*α* were decreased significantly in FS and SNT-HD groups compared to the model group (FS: 22.17 ± 8.66 ng/L, *P* < 0.05; SNT-LD: 25.61 ± 7.57 ng/L and SNT-HD: 23.94 ± 4.27 ng/L, *P* < 0.05 versus model group: 33.23 ± 5.78 ng/L). The levels of IL-1*β* were decreased significantly in serum (FS: 151.17 ± 16.62 ng/L, *P* < 0.01; SNT-LD: 170.91 ± 15.09 ng/L and SNT-HD: 170.8 ± 23.30 ng/L, *P* < 0.05 versus model group: 199.86 ± 25.44 ng/L) as well as in myocardial tissue (FS: 32.85 ± 3.64 ng/g, *P* < 0.01; SNT-LD: 37.32 ± 4.89 ng/g and SNT-HD ng/g, *P* < 0.05 versus model group: 41.56 ± 6.08 ng/g).

## 4. Discussion

In China, Chinese herbal medicine is widely used as an adjunct to biomedicine in treating MI [41]. Our previous studies indicated that SNT is suitable and safe for the animal model study and has the potential to improve early ventricular remodeling and cardiac function after MI [15, 16]. Pathological H&E staining showed that the IS values from the FS and SNT groups (23.91 ± 7.99 mm^2^, 31.25 ± 10.68 mm^2^ and 27.81 ± 10.33 mm^2^) were smaller than from the model group (38.04 ± 8.35 mm^2^). FS and SNT could decrease LVDs significantly in the FS and SNT-HD groups (FS: 3.81 ± 1.21 mm, *P* < 0.01; SNT-LD: 4.95 ± 1.95 mm and SNT-HD: 3.74 ± 1.47 mm, *P* < 0.01 versus the model group). FS and SNT could also decrease LVDd significantly only in the FS group (FS: 6.24 ± 0.72 mm, *P* < 0.05, SNT-LD: 5.37 ± 1.78 mm, and SNT-HD: 4.87 ± 1.47 mm versus the sham group). Echocardiography is the key diagnostic tool and was performed to assess LV function and volumes, valvular function, extent of myocardial damage, and to detect mechanical complications [42]. The results of our echocardiographic evaluation indicated that the rats in the SNT treated groups had an improved left ventricular function. The left ventricular ejection fraction (EF%) was significantly increased in all treatment groups compared with the model group (*P* < 0.05 and *P* < 0.01). Quality control of SNT by HPLC showed that no toxic diester-diterpenoid alkaloids of aconite were detected in the SNT decoction. The present study suggests that the Chinese herbal medicine SNT might play an important role in the treatment of MI and its associated inflammatory reactions.

Endothelin-1 (ET-1), a potent vasoconstrictor, is synthesized in the vasculature and myocardium by various cell types and is associated with the development of cardiac dysfunction. Nitric oxide (NO) plays an important role in the homeostasis of the cardiovascular system by regulating vascular smooth muscle cell contractility and myocardial oxygen consumption [21]. NO acts as a key contributor to vascular health due to its effects of limiting vascular inflammation, platelet aggregation, monocyte adhesion to endothelial cells, and abnormal smooth muscle cell proliferation. Endothelial dysfunction is connected to a decreased bioavailability of vasodilators, especially NO [22]. The levels of ET-1 in the plasma were decreased in all treatment groups but did not show significant differences among the groups in our experiments. The SNT-HD treatment group showed more decrease than other treatment groups. Yang et al. reported the regulating effect of SNT on blood pressure because it adjusts the expression levels of endothelin receptor-A and endothelial NO synthesis in the heart and the vasoactive marker levels (ET and NO) in the blood [43]. The NO levels of all treatment groups were increased. In comparison to the model group the SNT-HD group showed a significant difference (*P* < 0.05) in the NO level. NO was affected by the treatment with SNT at high doses.

Atrial natriuretic peptide (ANP) acts as a vasodilator which is released in response to increasing atrial filling pressures [23]. The most important factor governing ANP secretion is mechanical stretching of the atria, which occurs when extracellular fluid volume or blood volume is elevated. The release of ANP in disease states such as MI and HF appears to be related to both mechanical and cellular events [24]. The levels of ANP in the plasma of all treatment groups were lower than in the model group, but only the high dose group showed a significant difference (*P* < 0.05). ANP was also affected by the treatment with SNT at high doses. The examination of a larger number of subjects may be necessary to discover significant differences between the experimental groups.

Biochemical markers like collagen metabolites, proinflammatory cytokines, and matrix metalloproteinases are getting increasingly important in ventricular remodeling research and clinic cardiology. An ideal biochemical marker of clinical cardiology should be a prognostic indicator, should assist in the early diagnosis, reliably reflect the therapeutic response, and help in grading the risk associated with each stage of MI [38, 39]. CRP is an inflammatory biomarker which reflects the extent of myocardial necrosis and correlates with cardiac outcomes following AMI [6]. The inflammatory response and cytokines such as TNF-*α*, IL-1*β*, or IL-6 are increased soon after myocardial ischemic injury and can acutely regulate myocyte survival or apoptosis and trigger additional cellular inflammatory responses [7]. TNF-*α*, IL-1*β*, and IL-6 are not constitutively expressed in the normal heart [44]. There are robust upregulations of intramyocardial cytokines including TNF-*α*, IL-1*β*, and IL-6 mRNA expression in the infarct area and the noninfarcted myocardium after MI. In this study we could show that the levels of cytokines IL-6, IL-1*β*, and TNF-*α* and hs-CRP in rat serum and myocardial tissue to be decreased in the FS and the SNT treatment groups with a significant difference in the levels of IL-1*β*, TNF-*α*, and hs-CRP. SNT might have potential anti-inflammatory effects. This was described in the “Science of Prescriptions," a newly compiled practical English-Chinese library of traditional Chinese medicine [45] and is in agreement with various studies [46–50], which reported the pharmacological properties of ginger as an anti-inflammatory agent, the therapeutic function of cinnamon used for inflammatory diseases, fever, inflammation, chronic bronchitis, and for the improvement of blood circulation and the antigenotoxic and anti-inflammatory activities of licorice. To fully determine the anti-inflammatory effects of SNT thorough investigations should be performed including an evaluation of the number of infiltrating inflammatory cells and MI associated inflammatory cytokine levels in the future.

## 5. Conclusions

We evaluated the anti-inflammatory profiles of the Chinese herbal formula SNT, an ancient traditional medicinal formula using a rat model. Our data indicate that SNT could reverse ventricular remodeling and improve heart function. SNT has the potential to decrease the levels of hs-CRP and cytokines TNF-*α*, IL-6, and IL-1*β* after MI.

SNT decreased the expression of ET-1 levels in the plasma and increased the vascular active marker nitric oxide. In addition, the SNT high-dose treatment group decreased the expression levels of ANP in plasma significantly. These new findings will help us to develop more successful therapies including SNT for treating MI and its associated inflammatory responses.

## Figures and Tables

**Figure 1:** Quality control and toxicity evaluation of SNT by HPLC. (a) HPLC measurement of SNT. (b) The standard solution of diester-diterpenoid alkaloids: (1) mesaconitine, (2) hypaconitine, and (3) aconitine. mAU: milli absorption units.

**Figure 2:** Echocardiographic parameters. (a) Echocardiographic measurements of left ventricular dimension at end systole (LVDs), (b) left ventricular dimension at end diastole (LVDd), (c) left ventricular ejection fraction (EF), and (d) infarct size results.

**Figure 3:** Effects of SNT on ANP, ET-1 levels in plasma, and NO levels in serum. ANP (atrial natriuretic peptide) levels (a) and ET-1 (endothelin-1) levels (b) in plasma. NO (nitric oxide) levels in serum (c). ANP and NO levels of the SNT-HD group were significantly more different than those of the model group (*P* < 0.05).

**Figure 4:** Effects of SNT on the levels of inflammatory factors in serum and myocardial tissue. The hs-CRP levels (a) of the FS and the SNT treatment groups showed significant decreases in comparison to the model group (*P* < 0.01). The IL-6 levels in serum (b) were reduced in the FS and SNT treatment groups. The TNF-*α* levels (c) of the treatment groups were reduced. FS and the SNT-HD groups showed significant decreases in comparison to the model group (*P* < 0.05). The IL-1*β* levels in serum (d) were reduced in the FS and SNT groups (*P* < 0.01 and *P* < 0.05 versus model group, resp.). The IL-1*β* levels in myocardial tissue (e) were reduced in the FS and SNT groups and significantly in the FS and SNT-HD groups (*P* < 0.05 and *P* < 0.01, resp.) compared to model group.

**Table 1:** Composition of the Chinese herbal formula SNT.

Pin Yin	Chinese	Common	Latin	Amount/weight ratio
Zhi Fu Zi	*制附* *子*	Aconite	*Aconitum carmichaelii *	6
Rou Gui	*肉桂*	Cinnamon	*Cinnamomum cassia *	1
Gan Jiang	*干姜*	Ginger	*Zingiber officinale *	3
Jiu Gan Cao	*灸甘* *草*	Licorice	*Glycyrrhiza uralensis *	8

**Table 2:** The experimental rats groups. Drugs and decocts diluted with distilled drinking water were administered orally once a day for 30 days starting two days after induction of AMI.

Group	Sham	Model	FS	SNT-LD	SNT-HD
*N*	10	10	10	10	10
Operation	Sham	AMI	AMI	AMI	AMI
Oral administration	DW	DW	0.9 mg/kg	4.5 g/kg	13.5 g/kg

Sham: sham operated.

AMI: induced acute myocardial infarction.

DW: drinking water.

FS: fosinopril sodium (0.9 mg/kg).

SNT-LD: low dose of SNT (4.5 g/kg).

SNT-HD: high dose of SNT (13.5 g/kg).

**Table 3:** Echocardiographic parameters overview of ventricular remodeling effects.

	Sham	Model	FS	SNT-LD	SNT-HD	Remodeling effects (versus model)
LVDs (mm)	0.91 ± 0.20	6.44 ± 1.59**	3.81 ± 1.21^∗∗▲▲^	4.95 ± 1.95**	3.74 ± 1.47^∗∗▲▲^	↓
LVDd (mm)	3.29 ± 0.81	6.24 ± 0.72**	4.45 ± 1.28	5.37 ± 1.78	4.87 ± 1.47	↓
EF (%)	93.32 ± 2.94	55.48 ± 12.89**	78.03 ± 10.70^∗▲▲^	69.69 ± 13.91^∗∗▲^	77.83 ± 12.32^∗▲▲^	↑
IS (mm^2^)		38.04 ± 8.35	23.91 ± 7.99^▲▲^	31.25 ± 10.68	27.81 ± 4.91^▲^	↓

*P < 0.05, **P < 0.01 versus sham group; ^▲^ *P* < 0.05, ^▲▲^ *P* < 0.01 versus model group.

**Table 4:** Overview of vascular functional index marker expression levels in serum or in plasma ($\overset{-}{x}\pm s$).

	Sham	Model	FS	SNT-LD	SNT-HD	Expression levels (versus model)
ET (ng/L)	161.40 ± 13.95	171.09 ± 13.17	166.15 ± 9.01	166.74 ± 7.70	158.49 ± 9.97	↓
NO (µmol/L)	54.04 ± 11.88	48.18 ± 10.14	53.78 ± 6.24	53.06 ± 11.54	64.85 ± 8.74^▲^	↑
NO/ET	3.35	2.83	3.24	3.18	4.09^∗∗▲▲^	↑
ANP (ng/L)	250.00 ± 21.32	367.34 ± 43.20	222.26 ± 80.25	224.82 ± 80.19	189.05 ± 49.96^▲^	↓

ET and ANP were measured in plasma. NO was measured in serum.

**P < 0.01 versus sham group, ^▲^ *P* < 0.05, ^▲▲^ *P* < 0.01 versus model group.

**Table 5:** Overview of inflammatory factors and cytokines levels in serum and in myocardial tissue.

	Sham	Model	FS	SNT-LD	SNT-HD	Expression levels (versus model)
In serum						
hs-CRP (mg/L)	4.53 ± 0.66	6.71 ± 0.70**	5.02 ± 0.71^▲▲^	3.94 ± 0.61^▲▲^	3.97 ± 0.77^▲▲^	↓
IL-6 (ng/L)	204.17 ± 39.83	240.65 ± 27.80	210.60 ± 38.83	196.81 ± 22.68	202.55 ± 37.37	↓
TNF-*α* (ng/L)	23.38 ± 7.10	33.23 ± 5.78**	22.17 ± 8.66^▲^	25.61 ± 7.57	23.94 ± 4.27^▲^	↓
IL-1*β* (ng/L)	157.15 ± 17.34	199.86 ± 25.44**	151.17 ± 16.62^▲▲^	170.91 ± 15.09^▲^	170.8 ± 23.30^▲^	↓
In myocardial tissue						
IL-1*β* (ng/g)	29.73 ± 1.53	41.56 ± 6.08**	32.85 ± 3.64^▲^	37.32 ± 4.89	30.37 ± 1.91^▲▲^	↓

**P < 0.01 versus sham group; ^▲^ *P* < 0.05, ^▲▲^ *P* < 0.01 versus model group.
